# Effect of Midwives' Application of Intelligent Delivery Room Management System on Delivery Outcome

**DOI:** 10.1155/2022/4912053

**Published:** 2022-05-27

**Authors:** Xia Li, Ping Zhang, Yong Zhang, Gaiying Cui, Hui Du

**Affiliations:** Shijiazhuang Fourth Hospital, 16 Tanggu street, Chang'an District, Shijiazhuang City, Hebei Province, China

## Abstract

**Objective:**

To investigate the impact of midwives using an intelligent delivery room management system on the outcome of deliveries.

**Method:**

A total of 100 primiparas admitted to the department of obstetrics and gynecology of our hospital from January 2019 to June 2020 were selected as the research objects. They were randomly assigned to one of two groups: control or observation. The control group got standard obstetric care. On the basis of the control group, midwives in the observation group applied the intelligent delivery room management system for delivery management. The outcomes of childbirth, postpartum anxiety, and postpartum depression were recorded and compared between the two groups.

**Results:**

The observation group's first and second stages of labour were shorter than the control group's (*P* < 0.05), postpartum NRS score was lower than the control group's (*P* < 0.05), neonate Apgar score was higher than the control group's (*P* < 0.05), and the rate of vaginal delivery to caesarean section was lower than the control group's (*P* < 0.05). There was no statistical significance in prenatal S-AI scores between the observation group and the control group (*P* > 0.05). After delivery, the S-AI score of the observation group was lower than that of the control group, and the comparison result was statistically significant (*P* < 0.05). There was no significant difference in prenatal EPDS scores between the observation group and the control group (*P* > 0.05). After delivery, the EPDS score of the observation group was lower than that of the control group, and the comparison result was statistically significant (*P* < 0.05).

**Conclusion:**

Midwives may employ sophisticated delivery room management technologies to improve birth outcomes and reduce maternal anxiety and depression, and it is something that should be extensively promoted in clinic.

## 1. Introduction

Childbirth is a normal physiological process, and a constant and intense stressor, along with the delivery process, the maternal tension, anxiety, depression, and other adverse emotions increased sharply, and adverse emotions were correlated with the outcome of childbirth [1]. In obstetrics and gynecology, labor analgesia requires close observation. Turntable speed can also be slowed by prolonged work. Medical personnel are insufficient to address the demands of more women, resulting in the country's low natural birth rate [2, 3]. A clinic urgently needs a set of management system software to solve the problem of labor shortage in the delivery room. The system software can monitor the operation of the analgesic pump and physiological parameters of the pregnant women in real time. Electronic delivery record sheet can be realized, doctors can view all maternal actual labor process on a computer and can meet the needs of information, mobile monitoring function, electronic files, and so on [4, 5]. Midwives use an intelligent delivery room management system to optimise medical staff work efficiency, improve childbirth quality, control childbirth risk, and collect delivery room data management information [4, 6]. The use of the intelligent delivery room management system by midwives in our hospital from January 2019 to June 2020 had a positive impact on the delivery outcome, according to this study. The following is the report:

The paper's organization paragraph is as follows: the materials and methods is presented in Section 1.  Section 2 discusses the experiments and results. Finally, in Section 3, the research work is conclude with discussion.

## 2. Materials and Methods

### 2.1. General Information

A total of 100 primiparas admitted to the department of obstetrics and gynecology of our hospital from January 2019 to June 2020 were selected as the research objects. It had been approved by the Ethics Committee of our hospital. They were randomly divided into a control group and an observation group. Control group: the average age was 24.68 ± 4.21 years from 20 to 34 years old; gestational weeks ranged from 35 to 41 weeks, with an average of 39.64 ± 0.78 weeks. Observation group: the average age was 25.10 ± 4.22 years from 21 to 35 years old; gestational weeks ranged from 36 to 41 weeks, with an average of 39.88 ± 0.72 weeks. There was no significant difference in maternal age and gestational age between the two groups (*P* > 0.05), which was comparable.

#### 2.1.1. Inclusion Criteria

Inclusion criteria are as follows: ① 36 to 41 weeks of gestation; ② pseudonatural vaginal birth; ③ single live births; ④ age 20-35 years old; ⑤ the puerpera and her family members signed the informed consent.

#### 2.1.2. Exclusion Criteria

Exclusion criteria are as follows: ① patients with pregnancy hypertension and diabetes mellitus; ② patients with insomnia, depression, and other serious mental disorders before pregnancy; ③ patients with communication difficulties; ④ other unsuitable candidates.

### 2.2. Methods

#### 2.2.1. Control Group

Adopting routine obstetric management, that was, after entering the labor process, accompanied by the midwife, routine psychological support, breastfeeding guidance, and general guidance for the newborn.

#### 2.2.2. Observation Group

On the basis of the control group, with the use of midwives and intelligent delivery room management system for delivery management, intelligent delivery room management system from the perspective of the actual needs of the delivery room, covering the whole delivery process in the delivery room; it was necessary to support the real-time monitoring of the operation status of the analgesia pump, the real-time monitoring of the maternal physiological parameters, and the real-time monitoring of the portable monitoring equipment data, supporting the mobile viewing of medical staff, meeting the interaction data with HIS and other hospital information systems, and avoiding the generation of information islands [7]. The intelligent delivery room management system setted the delivery and delivery and postpartum rehabilitation in the same delivery room. Prepare Dulla ball, Dulla instrument, bean bag, and other birthing auxiliary supplies while equipped with a multipurpose electric bed, foetal monitor, low-frequency pulse postpartum rehabilitation equipment, first aid medications, narcotics, and other essential equipment during labour [8]. According to the home conditions of the puerpera, the ward environment was arranged; wardrobe, sofa, TV, 24 h hot water, and other necessary items for family life were added, and speakers were introduced to create an intelligent environment. Obstetricians, midwives, operating room nurses, neonatologists, nurses, and maternal family members collaborated during the delivery process to complete the perinatal management of the mother.  Figure 1 depicts the intelligent delivery room management system.

### 2.3. Observational Index

The outcomes of childbirth, postpartum anxiety, and postpartum depression were recorded and compared between the two groups.

#### 2.3.1. Delivery Outcome

The time of the first stage of labor, the time of the second stage of labor, the time of the third stage of labor, the number of cases of vaginal conversion to cesarean section, Apgar score of newborn, and labor pain were recorded in the two groups. Pain was assessed by numeral pain score (NRS) [9] at the first time after delivery; the pain intensity was expressed by 0~10 pain points, which were evaluated by the puerpera at the time of admission to the ward after delivery. The mean value was calculated by repeating twice.

#### 2.3.2. Postpartum Anxiety

The State Anxiety Questionnaire (S-AI) [10] was used to measure the state of maternal anxiety before and after 3 days. A total of 20 items were filled in by the parturients according to their own actual feelings. Each item was divided into 4 levels, which counted as 1-4 points. The higher the score, the heavier the anxiety level.

#### 2.3.3. Postpartum Depression

The Edinburgh Postpartum Depression Scale (EPDS) [11] was used to measure maternal depression at prenatal and postpartum 3 days. There were 10 items in total, and each item adopted a 4-level score of 0-3. The total score of each item was added into the total score, and the total score of >13 was classified as postpartum depression. The higher the score, the more severe the depression.

### 2.4. Statistical Methods

SPSS22.0 statistical software was used. The statistical data were compared by *χ*^2^ test of two independent samples. Two independent samples *t* or *t*′ test were used to compare the measurement data of normal distribution. Rank sum test was used to compare the measurement data of nonnormal distribution, and the test level *α* = 0.05.

## 3. Results

### 3.1. Results of Delivery Outcome

The time of the first stage of labor and the second stage of labor in the observation group were shorter than those in the control group (*P* < 0.05), postpartum NRS score was lower than control group (*P* < 0.05), Apgar score of neonates was higher than that of control group (*P* < 0.05), and the rate of vaginal delivery to cesarean section was lower than that of control group (*P* < 0.05). Results of delivery outcome are shown in Table 1.

### 3.2. Results of Anxiety Score

There was no statistical significance in prenatal S-AI scores between the observation group and the control group (*P* > 0.05). After delivery, the S-AI score of the observation group was lower than that of the control group, and the comparison result was statistically significant (*P* < 0.05). Results of anxiety score was shown in Table 2.

### 3.3. Results of Depression Score

There was no significant difference in prenatal EPDS scores between the observation group and the control group (*P* > 0.05). After delivery, the EPDS score of the observation group was lower than that of the control group, and the comparison result was statistically significant (*P* < 0.05). Results of depression score was shown in Table 3.

## 4. Discussion

In a set of system software, the intelligent delivery room management system integrates maternal analgesia with maternal and foetal physiological data. Support access to data information from a range of devices to satisfy the practical demands of obstetricians, anesthesiologists, and midwives at the same time. The software can also be based on warehouse conditions [12], optimize the system warehouse management workflow, and realize drug expiration query, material use instructions, and so on. It is convenient for the trainees to use it efficiently. It creates an electronic combat team and provides the function of multiangle and multilevel statistical analysis data to assist the commander in making decisions [13, 14]. Studies at home and abroad have reported that the incidence of anxiety and depression in pregnant women during pregnancy continues to increase. More than 50% of pregnant women show symptoms of anxiety or depression in the early and late stages of pregnancy, often showing extreme irritability, persistent fatigue and low mood, moodiness, and more tension, worry, and depression than before [15]. The physiological changes during pregnancy, social gestation pressure, postpartum fatigue, and complications that primipara face during pregnancy and delivery are likely to cause difficulty adapting to the role transition of novice mothers with no prior experience with pregnancy and delivery, an urgent demand for family support, and an easy to produce negative emotion [16]. Anxiety and depression during pregnancy not only directly damage the spirit and quality of life of pregnant women but also may develop into postpartum psychosis and bring long-term negative effects on the growth and development of infants [17]. The intelligent delivery room management system includes all living facilities and medical safety equipment, so that the parturient can feel warm during delivery and help the parturient to reduce the pain and stress reaction caused by negative emotions during delivery [18], prevent postpartum depression, and then reduce the risk of uterine weakness and prolonged labor, reduce the risk of neonatal asphyxia, and increase the natural birth rate. Because the medical equipment in use has safety risks, risk identification, risk assessment, and risk control are required [19]; the application quality evaluation of the analgesia pump should be strengthened in order to ensure the accuracy and reliability of the data collection of the intelligent delivery room management system [19].

Research in this study showed that the time of the first stage of labor and the second stage of labor in the observation group was shorter than those in the control group (*P* < 0.05), postpartum NRS score was lower than control group (*P* < 0.05), Apgar score of neonates was higher than that of control group (*P* < 0.05), and the rate of vaginal delivery to cesarean section was lower than that of control group (*P* < 0.05). There was no statistical significance in prenatal S-AI scores between the observation group and the control group (*P* > 0.05). After delivery, the S-AI score of the observation group was lower than that of the control group, and the comparison result was statistically significant (*P* < 0.05). There was no significant difference in prenatal EPDS scores between the observation group and the control group (*P* > 0.05). After delivery, the EPDS score of the observation group was lower than that of the control group, and the comparison result was statistically significant (*P* < 0.05).

To summarize, midwives using an intelligent delivery room management system can improve the result of labor, minimize maternal anxiety and depression, and is deserving of widespread clinical promotion.

## Figures and Tables

**Figure 1:** The intelligent delivery room management system.

**Table 1:** Results of delivery outcome.

Groups	Cases	Birth process time [M(Q_n_)∙h]			Apgar score		NRS	Normal delivery to cesarean section
		First stage	Second stage	Third stage	8-10	<8		
Control group	50	11.04 (0.75)	0.65 (0.13)	0.12 (0.02)	37	13	8.860 ± 0.280	14
Observation group	50	9.05 (1.32)	0.40 (0.17)	0.11 (0.03)	44	6	6.41 ± 1.170	6
Statistics		7.531	5.201	1.254	4.506		11.571	7.303
*P*		<0.050	<0.050	>0.050	<0.050		<0.050	<0.050

**Table 2:** Results of anxiety score.

Groups	Cases	S-AI	
		Before delivery	After delivery (3 d)
Control group	50	64.68 ± 1.650	60.31 ± 1.170
Observation group	50	65.03 ± 1.230	51.03 ± 1.610
Statistics		1.007	27.364
*P*		>0.050	<0.050

**Table 3:** Results of depression score.

Groups	Cases	EPDS	
		Before delivery	After delivery (3 d)
Control group	50	13.020 ± 2.340	9.020 ± 0.360
Observation group	50	13.140 ± 2.760	8.030 ± 0.760
Statistics		0.201	7.121
*P*		>0.050	<0.050

## Data Availability

The data used to support the findings of this study are included within the article.
